# Targeted non AR mediated smart delivery of abiraterone to the prostate cancer

**DOI:** 10.1371/journal.pone.0272396

**Published:** 2022-08-26

**Authors:** Abu Baker, Mohammad Khalid, Imran Uddin, Mohd Sajid Khan

**Affiliations:** 1 Nanomedicine & Nanobiotechnology Lab, Department of Biosciences, Integral University, Lucknow, India; 2 Department of Pharmacognosy, College of Pharmacy, Prince Sattam Bin Abduaziz University, Al-kharj, Saudi Arabia; 3 Department of Physics, SRM University-AP, Amaravati, India; 4 Department of Biochemistry, Aligarh Muslim University, Aligarh, India; Northwest University, UNITED STATES

## Abstract

Prostate cancer is the second-deadliest tumor in men all over the world. Different types of drugs with various delivery systems and pathways were developed, but no one showed prominent results against cancer. Meanwhile, nanoparticles have shown good results against cancer. Therefore, in the given study, citrate mediated synthesized gold nanoparticles (CtGNPs) with immobilized survivin antibodies (SvGNPs) were bioconjugated to the substantially potent drug abiraterone (AbSvGNPs) to develop as a combinatorial therapeutic against prostate cancer. The AbSvGNPs are made up of CtGNPs, survivin antibodies, and abiraterone. The selected drug abiraterone (Abira) possesses exceptionally good activity against prostate cancer, but cancer cells develop resistance against this drug and it also poses several severe side effects. Meanwhile, survivin antibodies were used to deliver AbSvGNPs specifically into cancer cells by considering survivin, an anti-apoptotic overexpressed protein in cancer cells, as a marker. The survivin antibodies have also been used to inhibit cancer cells as an immunotherapeutic agent. Similarly, CtGNPs were discovered to inhibit cancer cell proliferation via several transduction pathways. The given bioconjugated nanoparticles (AbSvGNPs) were found to be substantially effective against prostate cancer with an IC50 of 11.8 and 7.3 μM against DU145 and PC-3 cells, respectively. However, it was found safe against NRK and showed less than 25% cytotoxicity up to 20μM concentration. The as-synthesized nanoparticles CtGNPs, SvGNPs, and AbSvGNPs were characterized by several physical techniques to confirm their synthesis, whereas the immobilization of survivin antibodies and bioconjugation of Abira was confirmed by UV-visible spectroscopy, DLS, TEM, FTIR, and zeta-potential. The anticancer potential of AbSvGNPs was determined by MTT, DAPI, ROS, MITO, TUNEL ASSAY, and caspase-3 activity against DU145 and PC3 cells.

## 1. Introduction

The genome of cancer cells keeps changing with the advancement of the disease [1]. Cancer undergoes reorganization by remodeling its native signaling and function to rectify its intrinsic malfunctions for its rapid division and survival [2]. Cancer also maintains itself against drugs by re-routing signals and restoring homeostasis [2]. Prostate cancer is one of the most extensively recognized solid organ malignancies in males in the USA and the second most frequent worldwide. Moreover, metastatic castration-resistant prostate cancer (mCRPC) claims more than 30,000 lives per year in the USA [3]. Androgen receptor (AR) signaling [4] is the key cause of benign prostate hyperplasia (BPH), prostate cancer initiation, and progression of disease due to malfunctioned testosterone metabolism and its conversion to dihydrotestosterone in the presence of 5α reductase. For the last 75 years, androgen deprivation therapy (ADT), along with other therapies such as physical and chemical castrations, has been considered the first line of defense as a vanguard even at the advanced stage of disease [5, 6]. The risk of causing prostate cancer is increased by age, race, and family history [7, 8]. Although, PSA has replaced prostatic acid phosphatase (PAP) as a marker long back but due to a few shortcomings including severe inaccuracy for advanced-stage disease [9] certain new and advanced biomarkers, such as Select MDx (high accuracy for high-grade PCa), PHI, 4K, ExoDx, Mi-prostate score, PROGENSA PCA-3, prostate-specific membrane antigen, and survivin have been developed to diagnose prostate cancer precisely [10]. The U.S. FDA has approved the six most successful drugs viz., docetaxel, sipuleucel-T, abiraterone, enzalutamide, cabazitaxel, and radium-223 [11] based on their successful performance in improving the survival rate against mCRPC. Despite these approved therapies the disease state remains lethal. Abiraterone (Abira), among the 6 approved therapies is principally an irreversible inhibitor of CYP17A1 and prevents the production of dihydrotestosterone (DHT) from testosterone, and can directly bind to the AR and block its activity as a ligand-dependent transcription factor which leads to a frequent decline in prostate-specific antigen (PSA) and prolongs survival [12]. In the prostate cancer cell abira is converted into Δ4-abira (chief metabolite) in the presence of 3β-hydroxysteroid dehydrogenase (3βHSD). The Δ4-abira is a prominent inhibitor of DHT synthesis and antagonizes AR [13]. Another mechanism of abiraterone action seems to be even more complex, as it has been reported that it inhibits the pro-oncogenic TGFβ signals and induces apoptosis [14]. It is poorly soluble and has numerous side effects. Androgen receptor mutations are common in CRPC, and they are responsible for drug therapy failure. Other factors responsible for resistance are the generation of AR mRNA splice variants and mutations in several genes directly or indirectly associated with it [15]. However, not all tumors respond well to abira, and most tumors that respond eventually become resistant (in a widely variable duration) to abira. Clinical resistance to Abira is now frequently encountered in clinical oncology.

Nanotechnology is becoming routine in our daily life due to its dynamic development. EMA and FDA have approved various nano-based drugs with diverse formulations such as Caelyx®, Doxil®, Genexol-PM, Vyxeoes, Transdrug®, and Abraxane® are available in the market against cancer [16]. Lately, engineered gold nanoparticles have emerged as a prominent tool to treat cancer significantly [17]. Among metal and metal oxide nanoparticles, gold nanoparticles (GNPs) are non-toxic (up to 10^12^/ml) and highly biocompatible as one of the most successful delivery systems due to their easy tunability and synthesis [18, 19]. GNPs can deliver drugs into target cells using specific cell receptors and prevent the nonspecific interactions of drugs with other organs which make them highly biocompatible and nontoxic. The targeted anticancer therapy can also be used against cancer to block overexpressed receptors by antibodies [17, 20–22]. Survivin protein is an inhibitor of an apoptosis protein family (IAPs). It is involved in cell division dysregulation, and apoptosis [23]. It also supports tumor development by different pathways. Survivn protein also alters antitumor drug sensitivity. It is overexpressed in cancerous cells and least expressed in normal cells [24]. GNPs can directly enter the cytoplasm and nucleus, where they can degrade DNA and cause oxidation of proteins and fats. Therefore, in this study, non-AR mediated smart delivery of abiraterone to prostate cancer cells has been exploited through a nanomedicine comprising combinatorial therapeutics. The given nanomedicine exploited the intrinsic properties of GNPs to kill cancer cells along with abiraterone. The given nanomedicine was developed through bioconjugating the anti-prostate drug abiraterone to the survivin antibodies (SvAb) for cancer targeting over the surface of citrate mediated synthesized gold nanoparticles. The non-AR mode of action of abiraterone has been coupled and explained in terms of the synergistic action of various components of the proposed nanomedicines.

## 2. Material & methods

### 2.1. Materials

Survivin antibodies were procured from Invitrogen, abiraterone from TCI Chemicals (India) Pvt. Ltd., and Tetrachloroauric [III] acid (HAuCl_4_) from Sigma Aldrich (St. Louis, USA). The solutions were made before the experiment and stored in a dark place to keep them from any type of photochemical reactions.

### 2.2. Methods

#### 2.2.1. *Citrate mediated* synthesis of gold nanoparticles and immobilization of survivin antibodies

The citrate mediated synthesis of gold nanoparticles (C_t_GNPs) was performed by heating 1mM HAucl_4_ (3μl of 1 Molar stock) solution in 2.7 ml of double-distilled water at 100°C on a hot plate with the addition of 300 μl trisodium citrate solution (0.01 g/ml stock) at continuous stirring up to 400 rpm for 30 min. The reduction is fast as the reaction rapidly changes the color from colorless to grey to purple and then red.

Eventually, the immobilization of survivin antibodies over the surface of C_t_GNPs to get SvGNPs was performed by mixing 10μg/ml (10 μl of 1 mg/ml stock -PBS pH 7.4) survivin antibodies at room temperature with 1ml C_t_GNPs (1mM) nanoemulsion at slow stirring for 2 h at pH 7.6 which is more than the isoelectric point of survivin antibodies. Survivin antibodies’ immobilization prevents aggregation and provides stability to the emulsion of gold nanoparticles.

#### 2.2.2. Bioconjugation of SvGNPs with FDA approved anticancer drug abiraterone

The abira was immobilized over the surface of as-synthesized SvGNPs through covalent interaction by using 1-ethyl-3-(3 dimethyl aminopropyl)-carbodiimide (EDC) as the coupling agent. The coupling was achieved by mixing 50mM HEPES buffer (166 μl of 500 mM stock), 83 μg of abira (83 μl of 1 mg/ml stock), 1 ml of synthesized SvGNPs (1 mM), 185 μl of D.W. with 5 mM EDC (166 μl of 50 mM stock) in aliquots for 4–5 h at 30°C in total 1.66 ml of reaction mixture. The coupling was analyzed using UV-Visible spectroscopy after the completion of the reaction.

#### 2.2.3. Characterization of SvGNPs and AbSvGNPs

The SPR of C_t_GNPs was observed on a Shimadzu dual-beam spectrophotometer (model UV-1601 PC, Tokyo, Japan), operated at a resolution of 1 nm with gold nanoparticles at λ = 200–850nm wavelength range using a 1 cm quartz cuvette. UV-visible spectroscopy was also used to calculate the concentration of particles. Though UV/vis is simple, quick, and flexible, but advanced techniques are required to confirm the synthesis and conjugation by redshift. The mean particle size distribution of SvGNPs and AbSvGNPs was estimated by dynamic light scattering (DLS) using a Zeta sizer Nano ZS ZEN3600 apparatus (Malvern Instrument Ltd, Malvern, UK). It measures the size distribution and effective hydrodynamic diameter of the gold nanoparticles, and their aggregation was recorded at 25±0.1°C. Since, the study of zeta-potential was performed in an aqueous solution and different populations of the solution was checked. Therefore, the zeta-potential Smoluchowski approximation was used to calculate the zeta potential [25]. The size and morphology of SvGNPs and AbSvGNPs were examined under the transmission electron microscope (TEM) by using standard methodologies. TEM characterization carried out using an on Tecnai™ G2 Spirit BioTWIN, FEI, Hillsboro, USA operated at an accelerating voltage of 80 kV. At least 20 particles are taken to measure the size and shape of the TEM micrographs.

FTIR was done by forming individual films of each sample on a Si (111) substrate by using a drop of samples whereas water was evaporated by soft heating and FTIR spectra were observed on a Shimadzu FTIR8201 PerkinElmer Inc., Waltham, MA, USA apparatus in the reflectance scatter pattern at an assertion to get signal noise proportions of 4 cm^-1^. The bioconjugated film with 256 outputs was measured in the 400–4000 cm^-1^ range.

#### 2.2.4. Quantification of drug loading efficiency

The change in the absorption intensity of supernatant before and after the completion of the coupling reaction of abira with SvGNPs at 255 nm (λ_255_ nm) wavelength were used to calculate the percentage loading of abira. The percentage loading was calculated by substituting the observed values of A and B in Eq (1) [26].

$$Percentage\;loading\;of\;abiraterone\;on\;SvGNPs=\left(\frac{A-B}{A}\right)\times 100$$ (1)

where A- absorbance intensity of total amount (50 μg/ml) of abira added at the beginning of the reaction, B- absorbance intensity of abira (unbound) after completion of reactions [27].

The drug loading efficiency of abira was calculated by calibrating the standard graph at 255 nm in the concentration range of 20 to 100 μg/ml by using a UV-Vis spectrophotometer. The accurate amount of bioconjugated drugs can be obtained from Eq (2) after subtracting the unbound drug from the total amount of drug added.


$$Percent\;bioconjugation=\left(\frac{Amount\;of\;biocon\;jugated\;drug}{Total\;drug\;added}\right)\times 100$$ (2)

#### 2.2.5. Study of synergistic effects of SvGNPs and abiraterone drug

The synergism of two drugs having a different modes of action but their effects are directly proportional to their concentrations can be explained by Chou and Talalay method. Their collective effect can be explained by the “Combination Index”. The given investigation can be explained by calculating:

$$CI=\frac{d_{1}}{{ED50}_{1}}+\frac{d_{2}}{{ED50}_{2}}$$

$$=\left\{\frac{P}{(P+Q){ED50}_{1}}+\frac{Q}{(P+Q){ED50}_{2}}\right\}{ED50}_{c}$$

$$where,\;d_{1}=\left(\frac{P}{P+Q}\right){ED50}_{c}$$

$$d_{2}=\left(\frac{Q}{P+Q}\right){ED50}_{c}$$

Where d1 and d2 are the units of two different drugs used to get a 50% effect. ED50_c_ –Combined 50% inhibition; *ED*50_1_-IC_50_ of one drug and *ED*50_2_—IC_50_ of the second drug; Q and P- concentrations of two different drugs used to get combined 50% inhibition. CIA can explain the collective effectiveness as synergistic for CI < 1, for antagonistic CI > 1 and at CI = 1, the combination becomes additive [28].

#### 2.2.6. Cell culture

The prostate cancer DU145, PC3 cell line, and normal rat kidney (NRK) cell line were procured from National Centre for Cell Science (NCCS), Pune, India. RPMI medium was used to carry out the growth of DU145 and PC3 cells whereas DMEM-F12 medium was selected for NRK cells. Both the media were enriched with 12% sterilized FBS and 1.5% antibiotic-antimycotic solutions containing penicillin, streptomycin, and amphotericin B (Himedia, India, Ltd., Mumbai, India). The cells were incubated in a humidified chamber with 5% CO_2_ at 37°C.

#### 2.2.7. Determination of cell viability by MTT assay

The cytotoxicity of SvAb, C_t_GNPs, SvGNPs, pure abira, and AbSvGNPs was evaluated against DU145, PC3, and NRK cell lines by MTT assay [29]. The DU145, PC3, and NRK cells were seeded at a density of 5 ×10^3^ cells/well in 96 well plates at 37°C for 24 h in a humidified chamber with 5% CO_2_. Eventually, these adherent cells were treated with SvAb, C_t_GNPs, SvGNPs, Abira, and AbSvGNPs individually at different concentrations and incubated for 24h. Subsequently, treated cells were incubated with a 10 μl of 5 mg/ml MTT dye for 2 h at 37°C. The formazan crystal (purple colored) precipitates were obtained which were subsequently dissolved in 90 μl of dimethyl sulfoxide (DMSO). The absorbance of dissolved crystals of each well was measured at 570 nm on microplate reader (BIORAD-680 California, USA). The cell inhibition percentage was evaluated over the untreated cell. The IC-25, IC-50, and IC-75 values were evaluated by calibrating the graph between concentration and absorbance on Origin 6.0 Professional.

#### 2.2.8. Morphological analysis

Morphological analysis of C_t_GNPs, SvGNPs, Abira, and AbSvGNPs treated DU145, PC3, and NRK cells were done according to the method described elsewhere [30]. The cells were seeded at the density of 1.5 ×10^4^ cell/well for 24 h at 37°C in 24 well plates in a humidified chamber with 5% CO_2._ Eventually, a fresh medium supplemented with various dose concentrations (IC-25, IC-50, and IC-75) of C_t_GNPs, SvGNPs, Abira, and AbSvGNPs was added to further grow these cells for another 24 h in a humidified chamber with 5% CO_2_ at 37°C. Finally, morphological analyses of infected cells concerning the control cells were done using a phase-contrast microscope (Nikon ECLIPSE Ti-S, Nikon Corporation, Tokyo Japan).

#### 2.2.9. Measurement of intracellular ROS level

The production of intracellular ROS level in 24 H grown (1.5 x10^4^ cells/well) DU145 and PC3 cells after the treatment with various dose concentrations (IC-25, IC-50, and IC-75) of C_t_GNPs SvGNPs, Abira, and AbSvGNPs was measured in a 24 well plate by DCFH-DA method [31]. In brief, the treated cells were incubated with 10 μM of DCFH-DA and incubated for 30 minutes at 37°C in a humidified chamber with 5% CO_2_. The excess DCFH-DA was removed by gentle washing with 50 mM PBS at pH 7.2 and images were captured by using a magnifying lens (fluorescence microscope Evos FLC, Thermo Fisher Scientific, Waltham, MA 02451 USA) and Image J software was used to quantify the cellular fluorescence from fluorescence microscopy images.

#### 2.2.10. Study of nuclear condensation

In this study, the fluorescent dye DAPI was used to evaluate the nuclear condensation to confirm the apoptosis when DU145 and PC3, and NRK cells were treated with C_t_GNPs, SvGNPs, Abira, and AbSvGNPs following the method described elsewhere [32]. Briefly, DU145, and PC3 cells were seeded into 24 well plates at a density of 1.5 ×10^4^ cells/well and incubated at 37°C for 24 h. Eventually, C_t_GNPs, SvGNPs, Abira, and AbSvGNPs were incubated with these cells at IC-25, IC-50, and IC-75 concentrations for 24 h. In the next step, these cells were washed with cold PBS and fixed with 3.7% paraformaldehyde and subsequently, 300 nM DAPI was used to stain with 15 minutes of incubation at 37°C. The images of stained cells after the stipulated time were captured under an inverted fluorescence microscope (fluorescence microscope Evos FLC, Thermo Fisher Scientific, Waltham, MA 02451 USA). Finally, the cellular fluorescence of these cells was used to quantify the effect of different particles using Image J software.

#### 2.2.11. Mitochondrial membrane potential (ΔΨ m) estimation

The change in membrane potential of mitochondria was analyzed after treating DU145 and PC3 cells with C_t_GNPs, SvGNPs, Abira, and AbSvGNPs using Molecular Probes -M7512, Invitrogen kit according to the manufacturer’s protocol [33]. The experiment was carried out with the treatment of overnight grown DU145 and PC3 cells (1.5 ×10^4^ cells/well) in a 24-well plate with different doses (IC-25, IC-50, and IC-75) of C_t_GNPs, SvGNPs, Abira and AbSvGNPs for 24 h. Finally, the cells were stained with Mito Tracker Red (300nM) for 30 min in the dark, and images were captured using an inverted fluorescence microscope (fluorescence microscope Evos FLC, Thermo Fisher Scientific, Waltham, MA 02451 USA) at Texas red filter. Ultimately, the obtained cellular fluorescence was quantified under fluorescence microscopy using Image J software.

#### 2.2.12. TUNEL assay

The apoptosis in the cells were observed by terminal deoxynucleotides transferase-mediated UTP end labeling (TUNEL) staining (Invitrogen APO-BrdU™ TUNEL Assay Kit). DU145/ PC3 cells were grown in 24 well plates for 24 H in the density of 1.5×10^4^ cells/well and treated with C_t_GNPs, SvGNPs, Abira, and AbSvGNPs at IC-50 concentrations for another 24 h in a humidified chamber with 5% CO_2_ at 37°C and. Finally, the 4% paraformaldehyde was used to fix the cells and incubated in permeabilization solution (PBST) for 5 minutes. After permeabilization, cells were incubated with the DNA labeling solution (Reaction buffer, TdT enzyme, BrdUTP,) for 1 h at 37°C in the dark. Eventually, these cells were washed with rinse buffer for 5 minutes. Subsequently, an antibody staining solution (Alexa Fluor™ 488 dye-labeled anti-BrdU antibody and rinse buffer) was added and further incubated for 3 h at room temperature inside the humidified chamber and eventually, Propidium iodide/RNase staining buffer was added followed by incubation for 30 minutes at 37°C in the dark. Ultimately, 300 nM of DAPI stain was added and cells were observed under a fluorescence microscope (Evos FLC, Thermo Fisher Scientific, Waltham, MA 02451 USA). The apoptotic cells were determined by counting the total number of cells for fluorescein, Propidium iodide (PI), and DAPI.

#### 2.2.13. Evaluation of caspase-3 inhibition

To check the inhibition of caspase-3, approximately 1.5×10^5^ DU145 and PC3 cells were seeded for 24 H in a 6-well plate and subsequently transfected with IC-50 concentration of C_t_GNPs, SvGNPs, Abira, and AbSvGNPs for another 24 h. Caspase-3 activity assay was performed using Caspase-3/CPP32 Colorimetric Assay Kit (BioVision) according to the manufacturer’s instructions. Briefly, the treated cells were trypsinized and resuspended in 200 μl chilled cell lysis buffer and 2μL PMSF (1mM) on ice and constantly agitated at 4°C for 30 min. Further, these cells were centrifuged at 12000 rpm for 20 min to obtain protein in the supernatant. The total amount of protein was estimated by the Bradford method. The 100 μg from the obtained protein for each sample was mixed with 50 μl cell lysis buffer and 50 μl 2X Reaction Buffer (containing 10 mM DTT). Eventually, 5μl of 4mM DEVD-pNA-conjugated substrate was added to each tube, and each mixture was incubated at 37°C for 2 h. Ultimately, the absorbance at 405 nm by spectrophotometer was monitored using a 100 μl micro quartz cuvette. The increased CPP32 activity was determined by comparing these results with the level of the untreated control.

### 2.3. Statistical analysis

All statistical analyses were performed using the Origin 6.0 statistical software (USA), as described previously [34, 35].

## 3. Result

An appropriate delivery system enhances the effectiveness of the drug(s) strongly. Cancer is a disease that erupts due to rapid mutations (activation or loss of specific gene(s)) in a multistep process and with time these mutations accumulate in the cells. While newly arising cells of cancer will encounter different mutations and hence, generate a population of heterogeneous cells. Therefore, the best way to combat cancer is to use combinatorial drugs because heterogeneous cells require different therapeutics which can target different cells of tumors or cancer through diverse pathways. In the combinatorial system, one component potentiates the effect of others and in this way, the effective concentration of each component is reduced substantially to meet patient compliance. In the given study, an anticancer drug abira was selected to deliver to prostate cancer cells specifically. The abira was bioconjugated with survivin antibodies immobilized citrate mediated synthesized gold nanoparticles. This delivery system was found highly potential and inhibited the propagation of cancer cells at a substantially low concentration which convenes patient compliance (Scheme 1).

**Scheme 1:** Schematic representation of synthesis of abiraterone bioconjugated, survivin immobilized citrate gold nanoparticles (AbSvGNPs), their internalization (via caveolae-mediated, RTK, clathrin/ caveolin independent and simple diffusion mechanism) into prostate cancer cells and eventually, the production of ROS and role of each component of AbSvGNPs (i.e. C_t_GNPs, survivin antibodies and abiraterone).

### 3.1. Synthesis and characterization of C_t_GNPs and SvGNPs

In vitro synthesis of gold nanoparticles by reduction of the corresponding HAuCl_4_ is an apparent process. The citrate-mediated synthesis of gold nanoparticles depends on external conditions such as temperature and pH, which affect the quality and size of the nanoparticles. In this reaction, there are three significant parameters viz. concentration of gold chloride, the concentration of trisodium citrate & pH of the solution which regulates the size, shape, stability, and complete synthesis of citrate gold nanoparticle (C_t_GNPs). The synthesis of C_t_GNPs is initiated by the reduction of Au^+3^ to Au^0^ by citrate and the same citrate will function as a capping agent. The synthesis of GNPs was confirmed by using UV-visible spectroscopy (λ_Max_ -521 nm), transmission electron microscopy (15.6 nm), dynamic light scattering (46.3 nm) & zeta potential (-14.5 mV) [36].

After the complete synthesis of C_t_GNPs, functionalization of C_t_GNPs with survivin antibodies was done by directly adsorbing antibodies to the surface of particles through citrate-thiol and electrostatic interactions by exploiting citrate ions available on the surface of C_t_GNPs and amino/thiol groups of survivin antibodies. The immobilization was taken place at a pH slightly greater than the PI of survivin antibodies. The immobilization of survivin antibodies makes C_t_GNPs biocompatible. C_t_GNPs was found to show maximum absorption at 521nm (Fig 1A(a)) and functionalized nanoparticles (SvGNPs) at 524 nm (Fig 1A(a)). A slight red shift of the SPR peak is corresponding to the change in the refractive index of the surrounding media. The change in peak by 3nm is the confirmation of attachment of molecule(s) [37]. The hydrodynamic diameter (inorganic core with immobilized survivin antibodies and two layers of solvent) of SvGNPs was found to be 49.53 nm with a 0.229 particle distribution index (PDI) under DLS (Fig 1A(b)). This technique also determines different populations in the nanoemulsion [38]. Nanoemulsion of SvGNPs was found stable and showed good shelf life due to its overall anionic charge with −12.1 mV zeta potential (Fig 1A(c)). The stability of nanoemulsion at the low value of zeta potential can be explained by a low value of Hamakar constant [36]. TEM was used to measure the inorganic core (which was found to be ~17 nm) of SvGNPs with high resolution. The spherical-shaped particles were found to be monodispersed (Fig 1A(d)).

**Fig 1:** **A.** Characterization of SvGNPs under (a) UV-Visible spectra (b) Dynamic light scattering (c) Zeta potential and (d) Transmission Electron Microscopy. **B.** Characterization of AbSvGNPs under (a) UV-Visible spectra (b) Dynamic light scattering (c) Zeta potential and (d) Transmission Electron Microscopy.

### 3.2. Bioconjugation of abiraterone drug with SvGNPs and its characterization

The as-synthesized SvGNPs were bioconjugated with abira using the α-amino group of survivin antibodies exposed over the surface of NPs with the carboxylate group of abira drug. The binding was achieved through the EDC/NHS chemistry, which established a covalent bond (ie. a peptide bond) without the involvement of any spacer [39]. The UV-visible spectra representing surface plasmon resonance of AbSvGNPs and SvGNPs have been shown in Fig 1B(a). It was found that immobilization of survivin antibodies brought λ_max_ for SvGNPs from 521 nm to 524 nm and further, bioconjugation of abira drug shifted λ_max_ for AbSvGNPs from 524nm to 530 nm. The obtained spectra after each step was found to show broadening and decreased intensity The redshift in the absorbance spectrum by 6nm with broadening and decline in intensity confirmed the coupling [40] of the abira drug to SvGNPs (Fig 1B(a)). The hydrodynamic diameter of AbSvGNPs was found to be 88 nm with a 0.215 particle distribution index (PDI) under DLS (Fig 1B(b)). Also, AbSvGNPs emulsion was found to be highly stable with a zeta potential of -18.93 mV (Fig 1B(c)). Eventually, TEM was used to capture high-resolution images and the estimated average sizes of AbSvGNPs were obtained to be ~28 nm (Fig 1B(d)). The blur images with diminished sharpness of AbSvGNPs under TEM [41] also confirmed the binding of the drug. Finally, the spherical-shaped particles were found monodispersed under TEM.

### 3.3. FTIR spectroscopy of SvGNPs and AbSvGNPs

FTIR confirms and gives detailed information about ligands attached to the surface of nanoparticles. FTIR confirmed modifications in the secondary structure of native survivin antibodies, if any, after immobilization over the surface of GNPs. FTIR spectroscopy is used to study the conformational changes in proteins/antibodies by evaluating the change in characteristic protein peptide bonds (amide I/II) [42]. The given technique was further used to confirm the binding of abira with survivin antibodies immobilized on SvGNPs. Broadband at 3433 cm^−1^ (Fig 2(a)) ensured the presence of water molecules in the SvGNPs films. Further, the distinct peaks at 2077 cm^−1^ and 1637 cm^−1^ attribute the characteristic feature of survivin, a protein (Fig 2(a)). The peak broadening at 3408 cm^−1^ also ensured the coupling of abira with SvGNPs which corresponds to the–NH stretching present in the peptide bond with amide I and amide II [43]. Furthermore, The C-N stretching of aliphatic amines associated with peptide bond was confirmed by an extra characteristic peak at 1082 cm^−1^ which also makes bioconjugation confirm (Fig 2(b), 2(c)).

**Fig 2:** FTIR spectra of (a) SvGNPs, (b) Abiraterone, (c) AbSvGNPs, and (d) UV-Visible spectra of pure Abiraterone for drug loading efficiency and the data were expressed in mean ± SD of three experiments.

### 3.4. Quantification of drug loading efficiency

The loading percentage of abira on SvGNPs was ascertained by utilizing Eq (1). Furthermore, it was observed that bioconjugation of abira to SvGNPs is ~79.7% showing a proficient coupling of abira. Further, the quantification of bioconjugated abira to SvGNPs was also entrusted by UV-Vis spectroscopy (Fig 2(d)). The characteristic absorbance of the pure abira (at 255nm) [26] at 20, 40, 60, 80 100 μg/ml concentrations were used to calibrate the standard graph. It was found that ~78% bioconjugation of abira with SvGNPs took substantially high place.

### 3.5. Study of synergistic effects of SvGNPs and abiraterone drug

The synergism of SvGNPs and abira in AbSvGNPs was studied according to Chou Talalay by calculating their Combination Index (CI). The value of the CI against DU145 and PC3 cells was found to be 0.0118, and 0.0130, respectively. The CI value of less than one indicates that the effect of SvGNPs and abira is synergistic which also potentiates their effects and reduces effective concentration. The synergism will work well to get a good response of abira without any considerable side effects due to substantially low effective concentration which also goes well with patient compliance.

### 3.6. *In vitro* anticancer study of SvGNPs and abiraterone conjugated AbSvGNPs

The potential of AbSvGNPs was found to be significantly greater than pure abira against DU145 and PC3 cells while it did not show any cytotoxic effect against NRK cells. The inhibition increased with an increase in the concentration of C_t_GNPs, SvGNPs, Abira, and AbSvGNPs. The IC_50_ values of C_t_GNPs, SvGNPs, Abira, and AbSvGNPs against DU145 cells were found to be 225.7 μM, 100.58 μM, 36.7 μM, and 11.8 μM, respectively (Fig 3(b)–3(e)), and against PC3 cells they were found to be 128.8 μM, 106.8 μM, 24.8 μM, and 7.3 μM, (Fig 3(g)–3(j)). However, SvGNPs and AbSvGNPs did not show any significant cytotoxicity against NRK cells (Fig 3(m), 3(o)). On the contrary, C_t_GNPs and Abira were found to show cytotoxic effects against NRK cells with IC50 values of 307 μM and 27.8 μM, respectively (Fig 3(l), 3(n)). C_t_GNPs and SvGNPs showed substantially high cytotoxicity against prostate cancer cells. SvAb has a negligible effect against DU145, PC3, and NRK cells (Fig 3(a), 3(f), 3(k)). The effect of these particles were found maximum against the PC3 cell line although DU145 also received a good response.

**Fig 3:** The Cytotoxicity (dose dependent) study of SvAb, C_t_GNPs, SvGNPs, abira, and AbSvGNPs against DU145, PC3 prostate cancer cells and NRK normal cells. All the data were expressed in mean ± SD of three experiments.

### 3.7. Measurement of cytomorphological changes on DU145, PC3, and NRK cells

The morphological changes in DU145, PC3, and NRK cells were studied by incubating C_t_GNPs, SvGNPs, Abira, and AbSvGNPs at IC-25, IC-50, and IC-75 concentrations under phase contrast inverted microscope (Fig 4A–4C). The untreated (or control) cells were found to be unaffected with no change in native morphology after 24h of incubation (Fig 4A(a), 4B(a), 4C(a)). On the contrary, considerable changes in morphologies were found in DU145 and PC3 cells treated with AbSvGNPs at IC-25, IC-50, and IC-75 concentrations (Fig 4A(b), 4A(d), 4B(b), 4B(d)) whereas NRK cell didn’t show any significant changes in morphology after 24 h of exposure (Fig 4C(b)-4C(d)). Abira also created considerable deformations in the DU145, PC3 and NRK cells (Fig 4A(e)-4A(g), 4B(e)-4B(g), 4C(e)-4C(g)). C_t_GNPs and SvGNPs were also found to show considerable changes in DU145, and PC3 cells (Fig 4A(h)-4A(m), 4B(h)-4B(m)). But C_t_GNPs were also found to show significant morphological changes in NRK cells after treatment (Fig 4C(h)-4C(j)) while SvGNPs didn’t show any cytomorphological change (Fig 4C(k)-4C(m)) in NRK cells. After 24 h of treatment cells, were found to be detached, irregular, shrunk, and necrotic. Moreover, some detached and shrunk cells maintained their plasma membrane intact, showing that apoptosis had started.

**Fig 4:** **A.** Cytomorphological images after 24 h treatment of AbSvGNPs, abira, CtGNPs, and SvGNPs, at IC-25, IC-50, IC-75 against DU145 cell lines. Scale bar = 100 μm; 10X magnification. **B.** Cytomorphological images after 24 h treatment of AbSvGNPs, abira, CtGNPs, and SvGNPs, at IC-25, IC-50, IC-75 against PC3 cell lines. Scale bar = 100 μm; 10X magnification. **C.** Cytomorphological images after 24 h treatment of AbSvGNPs, abira, CtGNPs, and SvGNPs at IC-25, IC-50, IC-75 against NRK cell lines. Scale bar = 100 μm; 10X magnification.

### 3.8. Estimation of a generation of Reactive Oxygen Species (ROS)

The extent of intracellular ROS generation in the DU145 and PC3 cells upon interaction with C_t_GNPs, SvGNPs, Abira, and AbSvGNPs at IC-25, IC-50, and IC-75 concentrations were estimated by utilizing 5-(and6)- carboxy-2’,7’- dichlorodihydrofluorescein diacetate (DCFHDA) (Sigma-Aldrich) as an oxidation-sensitive fluorogenic marker of ROS in the viable cells (Fig 5A, 5B). The intensity of fluorescence was found to be directly proportional to the generation of ROS in the cells. The given analysis verified that AbSvGNPs treated DU145 and PC3 cells (Fig 5A(b)-5A(d), 5B(b)-5B(d)) were found to produce the greater intensities of fluorescence with respect to their controls (Fig 5A(a), 5B(a)). Intensities were found to increase while increasing the concentrations from IC-25 to IC50 but when the concentration was further increased to IC-75, the intensities were slightly decreased because at IC-75 almost 75% of cells got dead and only 25% of cells were able to produce fluorescence being in high-stress condition. Therefore, overall intensities at IC-75 were observed too much lower than at IC-25 and IC-50. Likewise, Abira treated DU145 and PC3 cells (Fig 5A(e)-5A(g), 5B(e)-5B(g)) were found to create remarkable fluorescence and C_t_GNPs, SvGNPs (Fig 5A(h)-5A(m), 5B(h)-5B(m)) treated cells were observed to emit brilliant fluorescence with defaced morphological structures due to elevated disrupting impact in the compactness of plasma membrane caused by ROS produced, though untreated cells did not show any consideration fluorescence and held their native morphology. The cytotoxicity impacts may apply through the generation of oxidative pressure and apoptosis with a possible association of overproduction of reactive oxygen species (ROS). Quantification of fluorescence using Image J software was used to quantify the fluorescence and it was also found that potentially AbSvGNPs generated a greater amount of fluorescence than C_t_GNPs, SvGNPs, Abira, and untreated cells at their respective IC-25, IC-50, and IC-75 concentration (Fig 5C(a), 5C(b)).

**Fig 5:** **A.** Images showing DCFDA staining under phase contrast microscope after 24 h treatment of AbSvGNPs, abira, CtGNPs, and SvGNPs at IC-25, IC-50, IC-75 concentration against DU145 cell lines. Scale bar = 50 μm; 20X magnification. **B.** Images showing DCFDA staining under phase contrast microscope after 24 h treatment of AbSvGNPs, abira, CtGNPs, and SvGNPs at IC-25, IC-50, IC-75 concentrations against against PC3 cell lines. against PC3 cell lines. Scale bar = 50 μm; 20X magnification. **C.** The evaluation of intensity of ROS generation in (a) DU145 and (b) PC3 cells after treating with CtGNPs, SvGNPs, abira, and AbSvGNPs at their respective IC-25, IC-50 and IC-75 concentrations. After treatment level of ROS increases fold respectively as compared to the untreated cells in (c) DU145 cells, and (d) PC3 cells. All the data were expressed in mean ± SD of three experiments, *P < 0.05, **P < 0.01 and ***P < 0.001 as compared with their respective control.

Quantitative estimation of ROS showed that AbSvGNPs treated DU145 cells produced 5.19 and 7.74 fold ROS, after treatment with IC-25 and IC-50 concentration, respectively while in PC3 cells ROS levels increased to 2.28 and 2.82 fold with respect to the control after treatment at IC-25 and IC-50, respectively. However, IC-75 treated DU145 and PC3 cells were found to produce a decreased level of ROS and it was estimated to be 7.28 and 2.32 fold, respectively due to a decrease in the number of live stressed cells after treatment. Likewise, C_t_GNPs, SvGNPs, and Abira treated DU145 and PC3 cells were observed to produce an increased level of ROS with respect to their controls (Fig 5C(a), 5C(d)). Hence the high level of ROS in AbSvGNPs treated DU145 and PC3 cells was estimated due to site-directed delivery of abira with the help of survivin antibodies as compared to native Abira. The overexpressed survivin in the prostate cancer cells plays an ideal target which could be targeted with the help of survivin antibodies.

### 3.9. Analysis of changes in nuclear morphology

The mechanism of cellular uptake and internalization of AbSvGNPs was additionally assessed by utilizing a fluorescent dye (4’, 6-diamidino-2-phenylindole) DAPI (Fig 6A, 6B). The C_t_GNPs, SvGNPs, Abira, and AbSvGNPs treated with DU145, and PC3 cells at IC-25, IC50, and IC-75 concentrations were incubated for 24 h at 37°C in a humidified chamber with 5% CO_2_ and stained by DAPI dye. The AbSvGNPs treated DU145, and PC3 cells were undergone into apoptosis and displayed extended cell membrane perforation; which achieved condensed chromatin and dark blue fluorescent consolidated nucleus (Fig 6A(b)-6A(d), 6B(b)-6B(d)) when judged against untreated cells (Fig 6A(A), 6B(A)). The abira treated positive control cells were also found distinctively fluorescent like NPs treated cells (Fig 6A(e)-6A(g), 6B(e)-6B(g)). The C_t_GNPs and SvGNPs also elicited apoptosis into the treated cells (Fig 6A(h)-6A(m), 6B(h)-6B(m)). Nuclear condensation is the prompt and peculiar manifestation of cytotoxic repercussions caused by stress. Image J software was used to quantify the fluorescence and it was found that AbSvGNPs treated cells created more intense fluorescence than C_t_GNPs, SvGNPs, Abira, and untreated cells at their respective IC-25, IC-50, and IC-75 concentrations (Fig 6C(a), 6C(b)). Quantitative results showed that the cellular apoptosis of AbSvGNPs increased to 1.94, 2.34, and 2.42 fold of the control level after treatment with IC-25, IC-50, and IC-75 concentrations, respectively in DU145 cells while in PC3 cells cellular apoptosis increased to 2.51, 3.62, 3.78 fold of the control level after treatment with IC-25, IC-50, and IC-75, respectively. Likewise, in C_t_GNPs, SvGNPs and Abira cellular apoptosis levels increased to many folds of the control level in DU145 and PC3 cells as shown in Fig 6C(c), 6C(d). Hence the high level of cellular apoptosis in AbSvGNPs treated DU145 and PC3 cells as compared to native Abira due to the increased efficacy of Abira when bioconjugated to SvGNPs.

**Fig 6:** **A.** Images showing DAPI staining under phase contrast microscope after 24 h treatment of AbSvGNPs, abira, CtGNPs, and SvGNPs at IC-25, IC-50, IC-75 concentration against DU145 cell lines. Scale bar = 50 μm; 20X magnification. **B.** Images showing DAPI staining under phase contrast microscope after 24 h treatment of AbSvGNPs, abira, CtGNPs, and SvGNPs at IC-25, IC-50, IC-75 concentration against PC3 cell lines. Scale bar = 50 μm; 20X magnification. **C.** The evaluation of DAPI stain cellular Apoptosis in (a) DU145 and (b) PC3 cells after treating with CtGNPs, SvGNPs, abira, and AbSvGNPs at their respective IC-25, IC-50 and IC-75 concentrations. After treatment cellular apoptosis increases fold respectively as compared to the untreated cells in (c) DU145 cells, and (d) PC3 cells. All the data were expressed in mean ± SD of three experiments, *P < 0.05, **P < 0.01 and ***P < 0.001 as compared with their respective control.

### 3.10. SvGNPs and AbSvGNPs disrupted mitochondrial membrane potential in DU145 and PC3 cells

The mitochondrial-derived apoptosis is elicited with the release of cyt-c after depletion of mitochondrial membrane potential (ΔΨm). The depletion in mitochondrial membrane potential ΔΨm after treating DU145, and PC3 cells at IC-25, IC-50, and IC-75 concentration of AbSvGNPs, abira, CtGNPs, and SvGNPs was examined by a specific dye Mito Tracker Red CMX Ros. The decrease in intensity of fluorescence was observed after treatment which signifies the decrease in ΔΨm as shown in (Fig 7A, 7B). The effect of AbSvGNPs, abira, CtGNPs, and SvGNPs on ΔΨm was found to be dose-dependent and it decreased in DU145 and a PC3 cell line with the increase in concentrations of AbSvGNPs, abira, CtGNPs, and SvGNPs (Fig 7A, 7B). Image J software was used to quantify the fluorescence of treated cells and it was found that AbSvGNPs generated less fluorescence than C_t_GNPs, SvGNPs, Abira, and untreated cells at their respective IC-25, IC-50, and IC-75 concentrations (Fig 7C(a), 7C(b)). Quantitative results showed that the ΔΨm of AbSvGNPs treated DU145 cells decreased by 5.5, 4.5, and 2.0 fold as compared to control at IC-25, IC-50, IC-75 concentration, respectively while in PC3 cells ΔΨm decreased by 5.7, 4.5, 3.0 fold in comparison to the control after treatment with IC-25, IC-50, IC-75, respectively. Likewise, in C_t_GNPs, SvGNPs, and Abira treated DU145 and PC3 cells ΔΨm decreased to many folds as compared to the control as shown in (Fig 7C(c), 7C(d)). Hence the high level of ΔΨm in AbSvGNPs treated DU145 and PC3 cells as compared to native Abira was due to the increased efficacy of Abira when bioconjugated to SvGNPs.

**Fig 7:** **A.** Images showing a Mitotracker Red CMXROS staining under phase contrast microscope after 24 h treatment of AbSvGNPs, abira, CtGNPs, and SvGNPs at IC-25, IC-50, and IC-75 concentration against DU145 cell lines. Scale bar = 50 μm; 20X magnification. **B.** Images showing a Mitotracker Red CMXROS staining under phase contrast microscope after 24 h treatment of AbSvGNPs, abira, CtGNPs, and SvGNPs at IC-25, IC-50, and IC-75 concentration against PC3 cell lines at Scale bar = 50 μm; 20X magnification. **C.** The evaluation of loss of mitochondrial membrane potential (ΔΨm) in (a) DU145 and (b) PC3 cells after treating with CtGNPs, SvGNPs, abira, and AbSvGNPs at their respective IC-25, IC-50 and IC-75 concentrations. After treatment mitochondrial membrane potential (ΔΨm) decreases fold respectively as compared to the untreated cells in (c) DU145 and (d) PC3 cells. All the data were expressed in mean ± SD of three experiments, *P < 0.05, **P < 0.01 and ***P < 0.001 as compared with their respective control.

### 3.11. Detection of AbSvGNPs induced Apoptosis by the TUNEL assay

To detect DNA degradation during the late stages of apoptosis TUNEL assay has been intended. In this method ruptured single or double-stranded DNA blunt end-labeled by TdT. TUNEL assay results confirmed the apoptotic effect of AbSvGNPs, abira, CtGNPs, and SvGNPs treated DU145 and PC3 cells at their IC-50 concentrations (Fig 8A, 8B). Apoptotic cells were observed by TUNEL and fluorescence green; while necrotic cells were detected by the red-fluorescent stain of propidium iodide. The number and green fluoresce of TUNEL-positive apoptotic cells were found to increase significantly in AbSvGNPs treated DU145 and PC3 cells when contrasted with the untreated cells. The green fluorescent intensity was noticed to increase in AbSvGNPs treated DU145 cells as compared to PC3 cells which assured that the pro-apoptotic effect was higher in DU145 cells as compared to PC3 cells. However, it was found that red fluorescence was increased in PC3 cells as contrasted to DU145 cells which assured that PC3 cells had cell cycle arrest and necrosis effects as compared to DU145 cells. Based on these results, it could be concluded that necrosis is more prevalent over apoptosis in C_t_GNPs, SvGNPs, Abira, and AbSvGNPs treated PC3 cells at IC-50 concentration as compared to Du145 cells.

**Fig 8:** **A.** Prostate cancer DU145 were treated with AbSvGNPs, abira, CtGNPs, and SvGNPs at IC-50 concentration for 24h and then labeled with DAPI, TUNEL and PI solution images. Scale bar = 50 μm; 20X magnification ation. **B.** Prostate cancer PC3 were treated with AbSvGNPs, abira, CtGNPs, and SvGNPs at IC-50 concentration for 24h and then labeled with DAPI, TUNEL and PI solution, images. Scale bar = 50 μm; 20X magnification ation. **C.** Activation of caspase 3 in CtGNPs, SvGNPs, abira, and AbSvGNPs treated (a) DU145 cells and (b) PC3 cells at IC-50 concentrations. All the data were expressed in mean ± SD of three experiments, *P < 0.05, **P < 0.01 and ***P < 0.001 as compared with their respective control.

### 3.12. AbSvGNPs induced activation of caspases-3 in prostate cancer DU145 and PC3 cells

Investigation of caspase-3, whether it plays any role during C_t_GNPs, SvGNPs, Abira, and AbSvGNPs induced apoptosis in DU145 and PC3 cells. Caspases are the key players of apoptosis and they execute the systematic degradation of selective cellular proteins after receiving a proper signal. The activation of caspase-3 is cyt-c mediated and it downstream the signals effectively Therefore, we dogged the activity in treated and untreated control cells. A significant induction of caspase-3 activities was observed in C_t_GNPs, SvGNPs, Abira, and AbSvGNPs treated DU145 and PC3 cells at IC-50 concentrations when incubated for 24 h at 37°C in a humidified chamber with 5% CO_2_ (Fig 8C(a), 8C(b)). Caspase-3 activity was significantly increased by 0.007, 0.008, 0.023, and 0.042 times in DU145 cell (Fig 8C(a)) and 0.041, 0.043, 0.048, and 0.072 times in PC3 cells (Fig 8C(b)) as contrasted to untreated control when treated at IC-50 concentration of C_t_GNPs, SvGNPs, Abira, and AbSvGNPs, respectively. Similarly, exposure to AbSvGNPs to induce caspase-3 activity was found to be significantly higher in DU145 and PC3 cells. Thus, the results of the caspase-3 activity assay signified the involvement of both the extrinsic and intrinsic pathways of apoptosis in AbSvGNPs treated prostate cancer cells.

## 4. Discussion

Abira is well known AR inhibitor and works as an ADT agent. It inhibits metastatic castrate resistance to prostate cancer (mCRPC) by selectively inhibiting CYP17A1 (a member of the city-P450 superfamily of enzymes) in an irreversible manner [44]. However, in the given study the role of abira against AR-negative PC3 and DU145 cells has been investigated. The effect of abira on AR null cells has been reported somewhere else also [14, 45]. Though, the exact mechanism of action of abira other than AR inhibition has not been completely explored. The observation clearly stated that the abira caused DNA damage non specifically irrespective of the AR status of the cell lines [45]. This feature of abira made it an anti-cancer drug for other cancers also than prostate cancer. It was postulated that abira damaged DNA via bypassing AR signaling such as corticosteroid receptors [46]. Other studies also confirmed the AR independent action of abira where inhibition and alteration of pro-oncogenic TGFβ signals and apoptotic factors have been explained, respectively [14]. The proposed delivery of abira in combinatorial therapeutics (AbSvGNPs) also explained the AR independent mode of action of the drug synergistically with C_t_GNPs and survivin antibodies. This system was found to produce IC_50_ at 11.8 and 7.3 μM against DU145 and PC3, respectively (Fig 3) which is much lower than the pure form of abira. The low concentration of effectiveness must subside the effect of severe side effects [47]. Also, the nonspecific interaction of abira with DNA will not pose any threat to resistance development [48] against the drug [49]. Therefore, a combinatorial strategy was developed to overcome the resistance and side effects of abira with the addition of survivin antibodies and C_t_GNPs. All three components of the given bioconjugated nanoparticles AbSvGNPs were found to potentiate the effect of each other and worked well in a synergistic manner. The components were found able to decrease the effective concentrations of each other which definitely lower the side effects and resistance of the abira. The effectiveness of AvSbGNPs is more against PC-3 (having high metastatic potential) than DU-145 (having moderate metastatic potential) due to the absence of PTEN, a tumor suppressor gene in PC3 cells [50]. The C_t_GNPs were selected as a core of this delivery system because it inhibits [51] tumor growth and metastasis by negating MAPK-signaling, up-regulating E-cadherin, and down-regulating Snail, N-Cadherin, and Vimentin. Eventually, survivin antibodies were immobilized over the surface of C_t_GNPs to target prostate cancer cells specifically because survivin is overexpressed in all 60 types of cancer [52]. The expression of survivin increases with the progression of cancer, angiogenesis, metastasis [53], drug resistance [54], chemotherapy, and radiotherapy [55, 56]. It is also found to pose resistance in prostate cancer against several drugs [57–59]. Therefore, various strategies [60] have been proposed for the inhibition of survivin which includes inhibition of survivin expression by mRNA translation, chemical inhibitors, gene therapy, and immunotherapy [61, 62]. Interestingly, secreted exosomes having survivin on their surface encourage accumulation and internalization of AbSvGNPs in the prostate cancer cells [63]. The dynamic and micro-tubule network mediated charge independent nonspecific internalization of particles takes place with the activation of receptor tyrosine kinase (RTK) present on the cell membrane [64, 65]. Hence, C_t_GNPs would be able to halt RTK-mediated RAF-MEK-MAPK pathways to inhibit cell propagation and differentiation. Diffusion, an Arf6/Cdc42/Rhoa dependent, specific lipid, and cholesterol mediated internalization also contribute substantially [66]. These pathways were found to deliver AbSvGNPs into the cytoplasm of prostate cancer cells where C_t_GNPs interacted with mitochondrial and cell membrane NADPH oxidase to create a range of ROS and superoxides, respectively (Fig 5A–5C). This interaction was also found to cause depletion in mitochondrial membrane potential (Fig 7A–7C). Eventually, this interaction originated leakage of mitochondrial Ca^2+^ ions with the activation of Ca^2+^ associated enzymes. The activated enzymes ultimately produced potent oxidizing and nitrating non-radical species [67, 68]. Further, this interaction also caused leakage of cyt-c and hence, initiation of caspase-mediated apoptosis (Fig 8A–8C). The given chain reaction produced a ROS burst which deactivated NF-κB pathway [69]. Further, survivin polyclonal antibodies landed in the cytoplasm with AbSvGNPs stimulated apoptosis and autophagy after halting the action of cytosolic survivin [70]. Also, the abira landed in the cytoplasm with AbSvGNPs and would have interacted with glucocorticoid receptors [46]. Furthermore, cationic charge-mediated internalization of AbSvGNPs is caveolae-mediated endocytosis and contributed to the maximum amount of NPs internalization. The internalized AbSvGNPs fused with caveosomes or multivesicular body (MTV) and didn’t interact with lysosomes. This pathway not only prevented the Abira from degradation but also gave it a chance to arrive into other organelles. The as-formed caveosomes containing AbSvGNPs passed along with microtubules to the nucleus via ER [71]. The AbSvGNPs successfully delivered unaltered Abira into the nucleus where it interacted nonspecifically with DNA and caused substantial degradation (Fig 6A–6C). Also, survivin antibodies delivered by AbSvGNPs into the nucleus, interacted with nuclear survivin and destabilized the chromosome passenger complex (CPC) to prevent cell division and expression of p53 gene. Now, during advancing towards nucleus AbSvGNPs passed through endoplasmic reticulum (ER) where they disturbed membrane integrity of ER and activated isoforms of nitrogen monoxide (NO) synthase (Ca2+/calmodulin-dependent enzymes) and produced NO which may react with superoxide to form peroxynitrite [67, 68]. After reaching to nucleus, CtGNPs created ROS and generated free radicals which interacted with DNA nonspecifically and damaged it which could trigger various responses including cell cycle arrest, protein oxidation/aggregation, apoptosis or mutagenesis [72].

## 5. Conclusion

The given study proposes a combinatorial system against prostate cancer using the FDA-approved drug abira. This drug was delivered with two more anticancer agents, viz., C_t_GNPs and survivin antibodies, as a nano vehicle. C_t_GNPs, SvGNPs, and abira inhibited PC3 with IC50 128.83, 105.1, and 24.6 μM, respectively, whereas their IC_50_ was found to be 225.7, 100.58, and 36.7 μM, respectively, against DU145. Interestingly, AvSbGNPs checked half of the growth of DU145 and PC3 cells at 11.8 and 7.3 μg/ml, respectively_._ The components of the AbSvGNPs were found to be effective at much lower concentrations than their pure forms because each component acted against prostate cancer through different pathways, which ultimately ended in reducing the effective concentration of each other. Therefore, a multi-targeting combinatorial system has been developed against prostate cancer with great patient compliance.
